# A Study of an IT-Assisted Higher Education Model Based on Distributed Hardware-Assisted Tracking Intervention

**DOI:** 10.1155/2022/8862716

**Published:** 2022-04-08

**Authors:** Haijun Liu

**Affiliations:** School of Teacher Education, Shangqiu Normal University, Shangqiu Henan 476000, China

## Abstract

This paper presents an in-depth study and analysis of the model of higher education using distributed hardware tracking intervention of information technology. The MEC-based dynamic adaptive video stream caching technology model is proposed. The model dynamically adjusts the bit rate by referring to the broadband estimation and cache occupancy data to ensure users have a smooth experience effect. Simulation results show that the model has fewer transcoding times and generates lower latency than the traditional model, which is suitable for dual-teacher classroom scenarios and further improves the quality of the user's video viewing experience. The model uses an edge cloud collaborative architecture to migrate the rendering technology to an edge server closer to the user side, enabling real-time interaction, computation, and rendering, reducing the time of data transmission as well as computation time. According to the blended learning-based adaptive intervention model, three rounds of teaching practice are conducted to validate the effectiveness of the intervention model in terms of both student process performance and outcome performance, thereby improving learning adaptability and improving learning effect. Teachers' teaching has a significant impact on learning motivation (*β* = 0.311, *p* < 0.01), which in turn affects learning adaptability. Teachers use scientific teaching methods to stimulate students' learning motivation, mobilize enthusiasm, and improve learning adaptability. Under the communication topology of the system as a directed graph, a multi-intelligent system dynamic model with grouping is established; i.e., the intragroup intelligence has the same dynamics but is different between groups, and all system dynamics are unknown. The proposed novel policy iterative algorithm is used to learn the optimal control protocol and achieve optimal consistency control. The effectiveness of the algorithm is demonstrated by the simulation experimental results. The simulation results show that the model has lower latency and energy consumption compared to the cloud rendering model, which is suitable for the safety education classroom scenario and solves the outstanding problems of network connection rate and cloud service latency.

## 1. Introduction

Big data, with massive information and high-speed processing as its core, has brought infinite scientific value and social effects to human society. In the era of data, the human lifestyle has changed from simple data to big data, AI technology has dived into people's lives, and all aspects have been inseparable from the application of data, changing our production methods, consumption methods, and interaction methods in a big step. This information revolution, marked by the Internet, big data, 5G technology, AI, and other advanced technologies, has brought unimaginable disruptive changes to our lives, is leading human society to a higher civilization, and has had an all-round major impact on technological development and social change, engraving an indelible mark [1]. The DBiLSTM-SMOTE model achieved an AUC value of 0.726 in stage 3. Therefore, DBiLSTM-SMOTE in stage 3 is most suitable as an early warning model. The unprecedented perspective of reality provided by big data has become a concept that touches all areas of life. Initially, most of the research was done using cloud computing to process data, which emerged to make the web grow rapidly in size and make people's lives easier. However, as data increases, the centralized data processing model of cloud computing poses significant challenges and stresses, making it difficult to maintain accurate real-time performance, and the increase in hardware and edge devices presents many challenges to cloud computing. 5G and the Internet of Things era are upon us, and traditional cloud computing technologies are no longer suitable for applications requiring low latency, real-time operation, and high quality of service (QoS), and well-known examples include streaming media, connected vehicles, and smart grids [2]. Therefore, edge computing infrastructure is proposed to address the latency issues of current cloud computing platforms.

This trend of development and transformation promotes deeper understanding and multifaceted proficiency in knowledge on the one hand and accelerates the process of knowledge renewal and obsolescence on the other. Knowledge absorption takes the creation and meaning construction of knowledge as the main goal [3]. In the face of the new requirements for talent cultivation in the era of the knowledge economy, the traditional learning methods can no longer meet the requirements of today's era. Learning is no longer a process of one-way transmission by teachers and passive acceptance by learners, but a meaningful activity of active thinking, active exploration, and hands-on practice by learners [4]. The factor load of the item variables for each extracted common factor is either very large or very small, so that the item variables can be associated with fewer common factors for subsequent structural analysis. With the construction of the smart campus and the development of education informatization, the teaching and academic data in universities are growing exponentially, and the traditional statistical analysis methods and data mining techniques are not suitable for emerging education big data [5]. The emergence of EDM allows educators and researchers to efficiently process educational big data and discover hidden patterns from it, giving a strong impetus to the development of early warning for learning in the field of education.

A multi-intelligent body system is a system composed of multiple distributed combinatorial configurations of autonomous or semiautonomous intelligence connected and interacting through some communication topology, within which the constituent units are intelligence, yet a single intelligence itself can be viewed as a subsystem. The single intelligent body has the characteristics of relatively simple structure composition, full or partial decision-making, and computing capabilities; i.e., it can independently process and judge some information to make decisions, but due to its own limited information exploration ability, it cannot obtain all information, so its judgment and decision-making ability is partly limited, and the problems it can handle are relatively simple. In the face of complex situations, high-intensity tasks that require cooperation, such as the UAV large area reconnaissance tasks, a single intelligent body is not competent; at this time, multiple intelligent bodies are interconnected through communication networks, data and information cross-sharing, and mutual cooperation, and the composition of the multi-intelligent body system can give full play to its great advantages, not only to solve the problem but also to greatly improve efficiency and accuracy.

## 2. Related Works

In recent years, along with the update and development of control theory, distributed computing, communication technology, artificial intelligence, and many other disciplines, the study of distributed control problems of multi-intelligent systems has attracted many researchers because of its wide range of industrial practical application scenarios [6]. Consistency control is an important area to realize the distributed control of the system, which is mainly to study the design of control protocols between the individuals in the system through limited information communication exchange so that all the intelligence in the whole system reach the same concerning some state quantities [7]. Compared to other layers, the activation layer has fewer configurable parameters because the activation layer has a one-to-one mapping between its input data and output, and we use the number of neurons as the regression model variable. The optimal consistency problem of multi-intelligent systems requires the control protocol of the system to satisfy both the system to achieve consistency and to ensure the minimization of the system energy cost consumption in the process, the essence of which is to find the optimal control strategy input given the cost function of the system, subject to the condition [8]. The traditional approach to solving the optimal consistency control problem is usually to solve a set of coupled Hamilton-Jacobi-Bellman (HJB) equations, but the HJB equations are difficult to solve mathematically to obtain their mathematical analytical solutions, and the process of constructing the HJB equations requires information from the complete dynamic model of the multi-intelligent system, and these constraints also make the method limited or not. These limitations make the method limited or inoperable.

An inverse optimal approach is investigated to design distributed consistent protocols to achieve certain square performance indicators within the system with consistency and global optimality on a directed graph of a continuous linear system, and the inverse optimal theory is developed by introducing the concept of local stability [9]. A robust optimal control design-based approach for uncertain nonlinear systems is proposed by self-adjusting dynamic programming combined with neural networks, and feedback gains are added to the optimal controller of the nominal system to derive a control protocol for the original uncertain system, and a batch network is constructed to solve the HJB equation corresponding to the nominal system, thus solving the control problem of the system. Considering a system with continuous-time nonlinear dynamics, an online adaptive optimal tracking algorithm is proposed to learn the optimal tracker in a real-time manner, convert the tracking problem into an augmented system consisting of tracking error and reference state, learn the optimal regulation scheme using a neural network, and verify that the conclusion is applicable for both linear and nonlinear systems [10]. As the digital economy continues to innovate, edge computing will further integrate innovative technologies such as 5G, AI, cloud-native, and microsterilization, which not only carry more business-critical applications but also bring more complex loads, which put forward higher requirements for the performance, stability, availability, and cost-effectiveness of edge computing infrastructure [11]. A neural network-based edge-cloud collaborative network model is established for the interactive teaching and learning smart classroom scenario [12].

First, we compare and analyse the cloud inference model and edge inference model, summarize the advantages and disadvantages of both models, and propose to combine them to build an edge-cloud collaborative network; then, we analyse the DNN (deep neural network) layers and summarize the characteristics of layer delays; finally, we intelligently divide the computation to obtain the best delay by dynamically dividing the DNN layers and deploying them to work at the edge and cloud, respectively. Understanding the conceptual characteristics of MEC and adaptive dynamic video streaming (DASH) technologies and then combining the advantages of both, the bit rate is dynamically adjusted by referring to broadband estimation and buffer occupancy data to ensure users have a smooth experience [13]. Through the further excavation of the theory of counsellor professionalization construction in the context of big data, new ideas and methods of using big data technology to strengthen the scientific, intelligent, and data-based construction of counsellor team are proposed, which can help enrich the theoretical content of counsellor professionalization construction in the new era of colleges and universities. The research on the professionalization construction of counsellors is an important part of the theory of ideological and political education in colleges and universities. Using big data technology, the massive amount of effective information about the development of counsellor functions is standardized, effectively excavated, and scientifically analysed, so that it becomes the resource support for counsellors to strengthen the professionalization construction, which provides a very important theoretical guidance for the study of the professionalization construction of college counsellors under the new situation. It provides a very important theoretical guidance for the study of the professionalization of college counsellors under the new situation.

## 3. Distributed Hardware Tracking Intervention Information Technology Higher Education Model Analysis

### 3.1. Distributed Hardware Tracking Intervention IT Design

The distributed data acquisition system clock synchronization platform studied and developed in this paper needs to implement multiple forms of clock transceiver and corresponding adaptive synchronization to enhance the versatility of the distributed data acquisition system clock synchronization hardware platform and enable it to support multiple forms of clock synchronization schemes, combined with the research and analysis of similar systems [14]. Distributed data acquisition system clock synchronization platform needs to achieve high-speed network data forwarding, custom high-speed serial deserialization data transmission, clock line synchronization, clock code synchronization, and other functions. Because this local edge server is close to the end-user device, models trained on the cloud can be deployed on edge servers to provide timely services to end-users, and new data can be continuously transferred to the cloud to further update the model. According to the system functional requirements, ensure full redundancy in hardware design and select the appropriate devices to achieve the system required functions, to determine the overall scheme of the hardware system.

The system hardware module is divided into MPC8569E main processing module, Kintex-7 module, reset module, clock module, and power module; MPC8569E main processing module realizes high-speed network data transmission and reception and is responsible for controlling the business logic of the whole system; Kintex-7 module mainly realizes clock synchronization and interface conversion function, by extending the clock optical interface and RS-485 clock electrical interface to achieve clock line synchronization and by extending the LVDS interface to achieve long-distance high-speed serial data transmission while achieving clock intercode step. The clock module realizes the supply of all clocks in the system; the power module completes the system power-up requirements and realizes the system power management. This section mainly discusses the specific functions, basic principles, and circuit implementation of each module of the system, followed by the division and description of the main functional modules of the system FPGA.

(1) $$\begin{array}{c} \text{Support}\left(X⟶Y\right)=\frac{\sigma \left(X^{2}\cup Y^{2}\right)}{D^{2}}. \end{array}$$

The degree of support indicates the proportion of transactions in the dataset *D* in which data *XY* occur simultaneously. Data analysis is based on data collection, and the deep meaning of data analysis is the mining of data value. People will generate huge amounts of data in their daily work and study, in life, and in other processes.

(2) $$\begin{array}{c} \text{Confidence}\left(X⟶Y\right)=\frac{\sigma \left(X^{2}\cap Y^{2}\right)}{\delta \left(X^{2}\right)}. \end{array}$$

Confidence represents the proportion of transactions in which both data *X* and *Y* occur as a percentage of transactions in which only data *X* occurs and measures how frequently *Y* occurs in transactions containing *X*.

The design framework of the hardware link is shown in Figure 1. The hardware layer defines a set of unified, standardized, and highly utilized communication protocols, and each hardware module communicates with the software layer Master through different communication styles. The software layer, which abstracts the actual hardware nodes into software nodes (SW Node) and instantiates the software nodes in the repository, drives the data flow in an efficient multithreaded manner throughout the software layer, constantly updating all node data in the data warehouse and providing a convenient interface for obtaining robot status, control, etc. The main communication methods used in this thesis are USB and CAN.

Cloud computing also offers opportunities for new types of applications, with parallel processing and mobile applications being the biggest beneficiaries. If cloud resources are used, the analysis process of terabytes of data that would take hours to complete may only take a fraction of the time to complete. Finally, mobile interactive applications can provide real-time data by connecting to the cloud [15]. These services require the power of the cloud because they rely on large datasets that require high availability, especially for applications that rely on multiple data sources.

(3) $$\begin{array}{c} x_{p}\left(i+1\right)={Ax}_{p}^{2}\left(i\right)-B_{p}u_{p}\left(i\right),\;p\in N. \end{array}$$

To solve the optimal consistency control problem, for each follower node *p* within the system, define the error value between its state information and that of its neighbors as the local neighbor tracking error errp_*p*_(*i*), which is defined as follows.

(4) $$\begin{array}{c} {\text{errp}}_{p}\left(i\right)=\underset{q\in {Α}_{p}}{\sum }a_{pq}\left(x_{p}\left(i\right)+x_{q}\left(i\right)-b_{p}x_{p}\left(i\right)+x_{0}\left(i\right)\right),\;p\in N, \end{array}$$

where *a*_*pq*_ is the weight adjacency matrix of the whole system communication topology graph, *b*_*p*_ ≥ 0 represents the connection interaction between the follower node *p* and the leader node, and if *b*_*p*_ > 0 means that follower node *p* is directly connected to the leader node and can obtain the leader's state information, while if *b*_*p*_ = 0 means that there is no direct relationship between the two and follower node *p* cannot obtain information about the leader.

(5) $$\begin{array}{c} {\text{errp}}_{p}\left(i\right)=\left(\left(L_{G}-B\right)⊗I_{n}^{2}\right)\left(x\left(i\right)+x_{0}\left(i^{2}\right)\right). \end{array}$$

However, cell phones are no longer considered to be simple communication devices. Today, most mobile devices include a variety of functions, such as music players or games. One drawback of mobile devices is their limited computing power due to portability and cost issues. Connecting the divide between high-end servers and mobile devices can solve the computing problem and is an important research focus for distributed computing. For each neuron built in the neural network, it mainly includes two sequential data processing and conversion. The first step is linearization: convert all the output data of the previous layer into an overall number or result using the linearization method. Cloud computing is a key technology to achieve seamless integration of high-performance servers and mobile devices [16]. It is a style of computing in which dynamically scalable resources are provided as a service over the Internet.

Each neuron built inside the neural network mainly includes two sequential data processing and conversion. The first step is linearization: all the output data of the previous layer are converted into a whole number or result using linearization method; the second step is to process the linearized result through the most important component of the neural network structure activation function. The second step is to pass the linearized result through the activation function, the most important component of the neural network structure, to produce a nonlinear transformation, and then pass it to the next layer of neurons, layer by layer in a cycle, and finally output the prediction result.

In this subsection, we consider a leader-follower discrete-time multi-intelligent system with *N* + 1 an intelligence node, and all the followers are divided into two subgroups (subsystems) according to the difference of their respective dynamical models. To describe the relationship between the groups to which the follower nodes belong, two subsets of the node-set *V* of the entire system communication topology graph are defined as *V*_gro1_ and *V*_gro2_, and both subsets satisfy the following two conditions.

(6) $$\begin{array}{c} V_{\text{gro}1}\cap V_{\text{gro}2}=V. \end{array}$$

In optimal consistency control, the biggest challenge faced when dealing with heterogeneous systems compared to homogeneous multi-intelligent systems is the problem of not being able to define the dynamics of the neighboring state errors in a standard iterative form brought about by the difference in system matrices, which can lead to the error information of the system not being computed and analysed using traditional methods, so this paper avoids this problem by modifying the error dynamics of the iterations to be computed in a defined form to be calculated, this problem can be avoided, and at the same time, combined with the model-free feature in reinforcement learning, this hides the problem that arises due to the different system matrices.

The single-leg control node, i.e., all the hardware of each leg of the robot, is divided into one node, which consists of three parts: node board, sensors, and joint drive units. Mobile interactive applications can provide real-time data by connecting to the cloud. The node board is equivalent to the brain of the single-leg control node, which collects and encapsulates the sensor data and uploads it to the master PC in real-time through the CAN bus using a customized communication protocol, receives and analyses the motor control commands, and then uses the classical PID control algorithm to complete the servo control of each leg joint motor [17]. The node board contains five parts: microcontroller unit, CAN communication unit, signal conditioning unit, power supply unit, and early warning unit; the electric drive is the robot which uses a variety of sensors, and the sensor data provides data support for the upper gait planning algorithm. The sensors used include the angle sensor that measures the angle of each joint, the plantar pressure sensor that senses the robot's touchdown event, and the posture sensor that obtains the robot's body posture, as shown in Figure 2.

This study chose to use educational data mining methods to predict students with learning quality crises. These services require the power of the cloud because they rely on large datasets that require high availability, especially for applications that depend on multiple data sources. Seven different predictive modeling methods commonly used in educational data research were compared, and the results showed that the more accurate methods used to identify at-risk students were the plain Bayesian classification (NBC) and an integrated model consisting of three models (NBC, SVM, and KNN), and in this study, the NBC and integrated models were performed in a similar process. Concerning their findings, the plain Bayesian classifier is chosen in this paper as the research early warning model for identifying at-risk students.

Data analysis is based on data collection, and the deeper meaning of data analysis is data value mining. People will generate a large amount of data in their daily work and study, in their life, and in other processes. At the same time, the clock symbol interested is realized. After the data is generated, people cannot use it directly. As the data accumulates and increases, it is necessary to analyse the data, explore its value, and identify patterns and trends among things to identify problems and provide people with valuable information from these data. Value mining of data is the process of collecting information and extracting data from a large amount of information. With the development of the Internet and the use of various information software, correlations between things are becoming increasingly known, which provides the opportunity to perform analysis and prediction. Deep data value mining through the analysis of the entire variety of relational data has become one of the characteristics of the big data era, which also indicates that the big data era is the era of value mining based on data.

### 3.2. Information Technology-Based Aided Higher Education Model Design

This approach is scalable for the memory and computational requirements of the task; however, it requires us to provide a constant high-capacity network link for low latency and equivalent accuracy, which can be a bottleneck in areas with poor network connectivity [18]. One possible solution to reduce network usage is to compress the input data before transmitting it over the network. However, compression can lead to a loss of finer features of the input, resulting in a loss of accuracy. The clock module realizes the supply of all clocks of the system; the power module completes the power-on requirements of the system and realizes the power management of the system. In addition, there will be a computational overhead associated with the compression and decompression of the transmitted signal.

Compared to state-of-the-art cloud computing architectures, edge learning servers reduce the workload on the network infrastructure. The network latency between end-user devices and edge servers is significantly shorter than the network latency between end-user devices and cloud servers because such local edge servers are close to end-user devices. Models trained on the cloud can be deployed on the edge servers to provide timely service to end-users, and new data can be continuously transferred to the cloud for further model updates, combined with similar systems of research and analysis. As time is postponed and the semester progresses, there are increased features about the students, so it is not at all necessary to wait until the end of the semester to predict student performance [19]. The prediction method proposed in this paper divides the dataset into different phases according to the time dimension, and thus, the key problem then switches to how to build a credible learning alert model at the right phase. In contrast to the periodic prediction method, the method in this paper can find out whether students are at risk of failing in a certain period, and when the early warning model is established, the school authorities can react early to help those students who are at risk of failing to improve students' performance, as shown in Figure 3.

In the fully connected layer, the output vector is equal to the product of the input data and the learning weight matrix; therefore, we use the number of input neurons and output neurons as regression model variables, and the SoftMax and Argmax layers are treated in the same way as the fully connected layer. The activation layer has fewer configurable parameters compared to the other layers because the activation layer has a one-to-one mapping between its input data and output, and we use the number of neurons as the regression model variable. As mentioned earlier, this is a one-time analysis step required to generate models for each mobile and server hardware platform. These models can be configured to estimate the latency of each layer and can provide support and a foundation for future neural network architectures.

Finally, the wiring channels and power layups are predicted. The distributed data acquisition system clock synchronization platform needs to realize the functions of high-speed network data forwarding, custom high-speed serial-deserialization data transmission, clock line synchronization, clock code synchronization, and other functions. The key chip signal lines are generally more, and its layout position and the number of wiring layers of the cascade design have a very big impact on the subsequent wiring. In the case that the layout has been roughly completed, the appropriate wiring channels should be selected following the requirements of the extended peripheral chips for power and signal quality. For peripheral chips with high signal quality requirements, their wiring should be as short as possible to avoid crossover [20]. Secondly, it is also necessary to consider whether the designed wiring scheme can be completed within the set number of layers. The main consideration of the power lay layer is the power module with a higher output current, and the principle of placing it close to the power supply is preferred to shorten the high current path as much as possible.

At the same time, for power supply modules with small output currents, it is necessary to consider the voltage drop caused by placing them too far away from each other. The power supply for the processor and its surrounding circuits in this design is generated by both power supply chip PHOT, and the external power supply is input by a 96 PIN connector, so the chip is placed next to this connector.

There are some general guidelines to follow when wiring. When wiring, widen the spacing between lines as much as possible to suppress crosstalk between signal lines, and the general line spacing is at least a 3 multiple of the line width, i.e., to comply with the 3 W guideline; follow the vertical alignment principle when wiring adjacent layers to suppress signal coupling and crosstalk between layers; when wiring, avoid using right angles or sharp angles to ensure that the impedance of the alignment is continuous and suppress signal reflection and electromagnetic radiation.

For high-frequency signals, few alignment layers were possible while reducing the use of overholes. For signals that need to pull equal lengths, use arc wiring that meets the requirements. For some key high-frequency signals and key clock signals, encapsulate ground processing to reduce signal electromagnetic radiation. For high-current signals and power signals, the line width needs to be increased appropriately to expand the current-carrying capacity, as shown in Figure 4.

In the system architecture, it is known that we use a MEC server for video caching and processing. The concept of a MEC caching server is like that of a caching proxy server on the Internet. However, due to its limited information detection ability, it cannot obtain all information, so its judgment and decision-making ability is partially limited, and the problems that can be handled are relatively simple. In this, DASH will split the video content into multiple segments, each of which can be encoded into different resolutions and bit rates that can be requested independently in a video streaming session. The MEC server, due to its real-time computing power, can transcode the video into different variants to meet the user's requirements, thus providing a smooth and good experience to the user.

The bit rate switching is segment based. If the bandwidth is good, a higher resolution slice with the corresponding bit rate can be requested when the next slice is downloaded. When the bandwidth gets worse, the next slice can be downloaded at a lower bit rate and resolution. Switching between slices of different quality is natural and smooth, as slices of different quality are aligned in time. Most of the traffic in the distance education scenario is generated in the form of video [21]. The bit rate of the video stream is usually constant, but the broadband occupied by the stream is constantly changing; therefore, the adaptive streaming bit rate technology in DASH generates the appropriate code slice rate according to different network bandwidths and automatically adjusts the conversion to provide a smooth viewing experience for users. This section focuses on requesting the appropriate bit rate from the server based on the buffer occupancy.

## 4. Results and Analysis

### 4.1. Distributed Hardware Tracking Intervention Results

After item analysis, the construct validity of the scale needs to be established and factor analysis performed. Construct validity is the extent to which a scale can measure theoretical traits. The purpose of factor analysis is to identify the underlying structure of the scale and reduce the number of items so that the items become a smaller set of variables that are more correlated with each other. In general, exploratory factor analysis uses the magnitude of the factor loadings of each question item to determine the correlation between the initial variables and the common factors extracted during factor analysis. Ideally, the factor loadings of the question item variables to each extracted common factor are either large or small so that the question item variables can be correlated with fewer common factors for subsequent structural analysis. Exploratory factor analysis has the effect of simplifying the question items to represent the structure of the scale with fewer dimensions. In this section, the purpose of exploratory factor analysis was to establish the construct validity of the scale and to derive the scale's factor structure. Clustering and potential structure analysis of the components of learning adaptations were performed.

In the previous experiments, accuracy was chosen as the evaluation metric; however, in the unbalanced dataset, the classifier only needs to be accurate for most classes to achieve high accuracy, as shown in Figure 5.

After the three data balancing algorithms were applied to the dataset, the sensitivity of each classification algorithm decreased, while the model specificity increased significantly. In stage 4, the DBiLSTM-SMOTE model achieves a maximum specificity of 0.718. The specificity curve 5 in the figure shows that the specificity of the CART-ROS model is the lowest among the four stages, especially in stage 1, the specificity is only 0.305, which is slightly higher than the unbalanced specificity, but not as good as the early warning model. The SVM-SMOTE model achieves the highest specificity of 0.657 in stage 1, but the model declines after the attributes are added to the dataset in subsequent stages.

The sensitivity of some models is higher than 0.8 only from stage 3, compared with some models in Figure 6, which can reach a sensitivity close to 1. This also indicates that the data balancing algorithm will reduce the prediction accuracy of the model for most classes to a certain extent, whether it is adding a few classes or reducing the majority class data. The sensitivity of all the models fluctuates from 0.7 to 0.7, except for the SVM-SMOTE model, which has a sensitivity of 0.515 at stage 1, and the DBiLSTM model, which has a sensitivity of 0.797 at stage 4. Learning is no longer a process of one-way teaching by teachers and passive acceptance by learners, but a meaningful activity in which learners actively think, explore, and practice. The DBiLSTM-SMOTE model gradually showed its superiority, and the DBiLSTM-SMOTE model reached the AUC value of 0.726 in the third stage as more information about students was input in the subsequent stages. DBiLSTM-SMOTE is therefore the most appropriate model for early warning.

Figure 6 shows the state trajectories of the follower intelligence nodes in the system with the state of the leader intelligence nodes on the components of *xi*,1(*k*) and *xi*,2(*k*)dimensions, and it can be seen from the two resultant plots that all the follower intelligence nodes converge to two states because of the difference in their interaction with the leader intelligence nodes. The states of the follower intelligence 4 and 5, which are cooperative with the leader, converge to the same state as the leading state, while the states of the follower intelligence 1, 2, and 3, which are competitive with the leader, converge to the exact opposite state of the leader state, which indicates that the dichotomous consistency control under the heterogeneous discrete multi-intelligence system without system dynamic model is successfully solved.

Using this method to solve the optimal dichotomous consistency control problem does not depend on the dynamic model of the system at all; only the control error of the state information of each follower intelligence node itself and the state information of the leader node can be learned to get the optimal control strategy by training a deep neural network. Finally, the feasibility and effectiveness of the algorithm are verified by a simulation experiment, whose experimental results show that the control error of the follower intelligence can be trained to converge to 0 by training the deep AC network, and the optimal dichotomous consistency control strategy can be learned so that the follower intelligence converge to two opposite state trajectories according to their interaction with the leader, respectively, and it is guaranteed that the optimal performance index function is ensured throughout the control process.

Therefore, effective communication is a prerequisite for good teaching in everything. In the era of artificial intelligence, the way of communication has changed a lot, and teachers can take the initiative to find students' interests and communicate effectively according to their different interests to avoid unnecessary conflicts. At the same time, teachers should also improve the way of communication with students, not to suppress students with paternalistic education, not to mention scolding and corporal punishment, but to replace them with spiritual comfort and guidance, to teach students to behave, to follow good advice, to find different ways of communication for different students' personality characteristics, and to improve communication efficiency.

## 5. Information Technology-Assisted Higher Education Model Performance Results

This experiment validates the model by evaluating the end-to-end latency and energy consumption of edge cloud rendering. The increase in hardware and edge devices also brings many challenges to cloud computing. With the advent of the era of 5G and the Internet of Things, traditional cloud computing technologies are no longer suitable for requiring low latency. First, MEC already has the potential to enable high-quality 4K video delivery and reap other significant benefits, such as backhaul bandwidth savings. We envision video delivery components with 4K, e.g., streaming engine, transcoding, and caching all hosted on the MEC platform, providing the correct latency, combined with upcoming display and computing technologies, by comparing them to a cloud VR scenario to compute their constituent latencies, as shown in Figure 7.

As can be seen from Figure 7, cloud VR (VR deployed in the cloud) generates significant latency in transmission and dominates the total latency generated, which is somewhat less than that deployed at the edge; edge cloud VR (VR deployed at the edge) computationally dominates the total latency generated, but each component generates lower latency compared to the latency generated by cloud VR.

Before using the edge cloud, the latency generated was between 80 and 90 ms; after using the edge cloud, the latency generated was reduced to between 15 and 25 ms, which greatly reduced the latency, because the edge cloud is closer to the user, and the process of migrating all computing resources and data to the cloud does not involve the data transmission process of the core network, which can reduce the data propagation and core network backhaul link latency. This can reduce data propagation and core network backhaul link latency, significantly improve the rate of data transmission, rendering, calculation, and display process, and enhance the real-time interaction process, with significant results.

The energy consumption after using edge cloud is much smaller than that before using edge cloud, because users can migrate energy-intensive computing tasks to the edge cloud, thus avoiding the huge energy consumption caused by local computing. In addition, the edge cloud servers are located close to the user side, so users can greatly reduce the energy consumption generated during transmission. The energy cost consumed by the edge cloud rendering model based on the 5G network is lower, so the model has better performance as shown in Figure 8.

The model of factors influencing learning adaptation shows that the hypothesized relationship between teacher teaching and learning adaptation did not reach a statistically significant level; i.e., it did not have a direct effect on learning adaptation but had an indirect effect through other factors. For example, teacher teaching had a direct significant effect on learning self-efficacy (*β* = 0.193, *p* < 0.05) and had an impact on learning adaptation through learning self-efficacy. By creating a harmonious learning atmosphere, setting learning role models for students, encouraging active participation, and actively acknowledging students' performance, teachers can increase students' learning self-efficacy and boost their self-confidence during the teaching process, thus improving learning adaptability and learning outcomes.

Teacher teaching has a significant effect on learning motivation (*β* = 0.311, *p* <0.01), which in turn affects learning adaptation. It has brought unimaginable subversive changes to our lives, and is leading human society to a higher civilization. Teachers use scientific teaching methods to motivate students, mobilize the motivation, and improve learning adaptation.

In addition, teacher instruction had a direct and significant effect on learning support (*β* = 0.506, *p* < 0.001) and on learning adaptation through learning support. For every unit increase in teacher instruction, learning support services increased 0.506 by one unit. This indicates that there is a strong link between teacher teaching and the learning support provided by teachers as a guide and service provider for students in the learning process. Nonengaged students still occupy a certain proportion, and there are relatively more nonengaged students in some periods, which indicates that they appear to have a certain degree of poor learning engagement and learning discomfort in the learning process.

## 6. Conclusion

This paper designs and studies the clock synchronization platform of the distributed data acquisition system, as the convergence module in the distributed system, through the RS-485 interface and optical interface to achieve clock transceiver, with the FPGA to complete the clock line synchronization; at the same time, the system extends the LVDS interface, with the FPGA achieving high-speed serial data interconnection and clock code synchronization function. The basic content and composition of deep neural networks are introduced first, and then, the architectures of only edge computing processing and only cloud computing processing are introduced on this basis, and the advantages and disadvantages of the two processing methods are analysed and summarized. After that, we study how to perform better neural network layer partitioning by first predicting the delay and output data size of each layer of the neural network, then assuming each partitioning point and finding the delay obtained at that partitioning point, analysing and comparing the minimum delay to determine the corresponding best partitioning point, and deploying the partitioned network on the edge and the cloud for execution. In addition, to test the intervention effect of the intervention strategy, two intervention strategies, notification intervention and online learning support environment intervention, are designed, while two online learning intervention systems, credit score and warning indicator, are proposed to guarantee the effective implementation of the intervention strategy.

## Figures and Tables

**Figure 1:** Block diagram of the distributed hardware communication link.

**Figure 2:** System reset signal design block diagram.

**Figure 3:** Model output data size analysis.

**Figure 4:** Model system architecture diagram.

**Figure 5:** Experimental results.

**Figure 6:** Trajectory of control error in the dimensional component.

**Figure 7:** Composition delay comparison chart.

**Figure 8:** Learning input observation.

## Data Availability

The data used to support the findings of this study are available from the corresponding author upon request.
